This article has been retracted.

# Efficacy of Gamma Globulin Combined with Azithromycin Sequential Therapy in the Treatment of RMPP and Its Effect on Th1/Th2 Cytokine Levels

**DOI:** 10.1155/2022/5162768

**Published:** 2022-07-20

**Authors:** Jie Qi, Fang Jia, Hui Tian, Shengmei Yang

**Affiliations:** Special Needs Ward, Shanxi Children's Hospital, Taiyuan 030013, China

## Abstract

**Objective:**

To investigate the efficacy of gamma globulin combined with azithromycin sequential therapy in the treatment of children with refractory mycoplasma pneumonia and its effect on Th1/Th2 cytokine levels.

**Method:**

From January 2021 to January 2022, 100 children diagnosed with refractory mycoplasma pneumonia were randomly divided into 2 groups (50 cases in each one), the control group was treated with azithromycin plus comprehensive basic treatment, and the treatment group was treated with combined treatment on the basis of the control group, gamma globulin therapy; the treatment effect and cytokine levels of the two groups were compared.

**Results:**

Th1, Th2, and Th1/Th2 before treatment were not significantly different between the two groups. Th1, Th2, and Th1/Th2 in the treatment group were significantly downregulated compared with those in the control group after treatment. The levels of IgG, IgA, and IgM in the treatment group were not significantly different from those in the control group before treatment but were significantly upregulated after treatment. IL-10, IL-6, and IL-2 levels were also significantly increased in the treatment group. The disappearance time of clinical symptoms such as fever, cough, and pulmonary rales in the treatment group was significantly shorter than that in the control group, and the cure rate in the treatment group was significantly better than that in the control group.

**Conclusion:**

The clinical effect of gamma globulin combined with azithromycin sequential therapy in the treatment of children with refractory mycoplasma pneumonia is remarkable, which can reduce inflammatory factors, improve patients' immunity, and promote disease recovery.

## 1. Introduction

Refractory Mycoplasma pneumoniae pneumonia (RMPP) mainly refers to mycoplasma pneumonia characterized by persistent fever, progressive aggravation of clinical symptoms, and related imaging manifestations after 1 week of standard macrolide therapy [1]. Acquired pneumonia with unknown clinical etiology changes rapidly, and extensive pulmonary inflammation can occur in a relatively short period of time, often accompanied by complications such as massive pleural effusion, pleural thickening, lung abscess, and pneumothorax. In more severe cases, children may develop bronchiolitis obliterans, atelectasis, and systemic inflammatory response syndrome, posing serious health risks [2]. At present, the treatment of refractory Mycoplasma pneumoniae pneumonia mainly adopts antibacterial, inhibiting overactive immune response and bronchoalveolar lavage, but the clinical efficacy is still poor [3]. In recent years, azithromycin is clinically combined with basic therapy. It has been reported that the pathogenesis of severe Mycoplasma pneumoniae pneumonia is related to cell-mediated immunity, and corticosteroid therapy may be effective. Intravenous immunoglobulin (IVIG) has been used as a potent immunomodulator for Kawasaki disease and other immune-mediated diseases [4]. Intravenous immune globulin can also be used to treat refractory Mycoplasma pneumoniae pneumonia. Therefore, this study is aimed at investigating the treatment options for refractory mycoplasma pneumonia in children.

## 2. Materials and Methods

### 2.1. Patients

From January 2021 to January 2022, 100 pediatric patients diagnosed with refractory mycoplasma pneumonia were randomly divided into 2 groups (50 cases in each). All patients in this study gave informed consent, and the patients themselves or their representatives signed the relevant consent forms. The details of the baseline data of the included subjects are summarized in Table 1.

### 2.2. Inclusion and Exclusion Criteria

The inclusion criteria for this study were (1) meeting the diagnostic criteria for refractory mycoplasma pneumonia in “Practical Internal Medicine” and (2) no related treatment was performed before inclusion in the study.

The exclusion criteria were (1) combined with other respiratory diseases, (2) related to malignant tumors and other diseases, and (3) suffering from mental illness or drug allergy.

### 2.3. Interventions

The children in the control group were treated with conventional treatment measures such as fever reduction, oxygen inhalation, atomization, cough relief, phlegm reduction, and azithromycin. Administer 10 mg/kg body weight on the first day, the maximum daily dose does not exceed 0.5 g, and on the 2nd to 5th days, administer oral 5 mg/kg body weight; the maximum dose does not exceed 0.25 g. Continue treatment for 2 weeks. The patients in the treatment group were given routine basic therapy at the same time, gamma globulin combined with azithromycin. The gamma globulin was dissolved in normal saline for intravenous infusion.

### 2.4. Observation Indicator

The clinical efficacy of the two groups of patients was compared. T lymphocyte factors Th1, Th2, and Th1/Th2; inflammatory factors IL-10, IL-6, and IL-2; and immunoglobulin levels IgG, IgA, and IgM were determined by commercial ELISA kits (Abcam, USA).

### 2.5. Statistical Analysis

The experimental data was analyzed by SPSS21.0 software (SPSS, Chicago, USA), the count data was analyzed by *χ*^2^ (%), the measurement value was analyzed by *t* test, and two-sided *P* < 0.05 was used to judge whether there was a statistically significant difference.

## 3. Results

### 3.1. Comparison of Th1, Th2, and Th1/Th2 between the Two Groups before and after Treatment

As shown in Table 2, Th1 (0.53 ± 0.15), Th2 (0.47 ± 0.13), and Th1/Th2 (1.41 ± 0.20) in the treatment group were compared with those in the control group Th1 (0.57 ± 0.16), Th2 (0.46 ± 0.14), and Th1/Th2 (1.43 ± 0.15) which had no significant difference (*t* = 2.019, 1.631, and 1.461; *P* = 0.245, 0.131, and 0.102). After treatment, Th1 (0.16 ± 0.14), Th2 (0.18 ± 0.07), and Th1/Th2 (0.39 ± 0.16) in the treatment group were lower than those in the control group Th1 (0.37 ± 0.2), Th2 (0.31 ± 0.06), and Th1/Th2 (0.58 ± 0.58 ± 0.18), and the difference was significant (*t* = 15.943, 12.005, and 13.325; *P* = 0.001, 0.005, and 0.005).

### 3.2. Comparison of Serum Immunoglobulin Levels between the Two Groups before and after Treatment

As shown in Table 3, before treatment, IgG (8.50 ± 1.40), IgA (1.40 ± 0.20), and IgM (1.50 ± 0.30) in the treatment group were compared with IgG (8.30 ± 1.60), IgA (1.20 ± 0.30), and IgM (1.50 ± 0.20) in the control group, and there was no significant difference (*t* = 1.568, 1.064, and 1.263; *P* = 0.712, 0.070, and 0.065). After treatment, IgG (11.20 ± 1.60), IgA (2.20 ± 0.30), and IgM (1.70 ± 0.10) in the treatment group were significantly higher than those in the control group in terms of IgG (9.50 ± 1.80), IgA (1.80 ± 0.40), and IgM (1.60 ± 0.30, *t* = 12.018, 11.935, and 10.881; *P* = 0.001, 0.003, and 0.001).

### 3.3. Comparison of Inflammatory Factors before and after Treatment in the Two Groups

After treatment, IL-10 (30.20 ± 5.23), IL-6 (40.52 ± 2.83), and IL-2 (30.61 ± 1.50) in the treatment group were significantly lower than those in the control group IL-10 (19.91 ± 5.40) and IL-6 (48.21 ± 1.50) and IL-2 (21.20 ± 2.41), and the difference was significant (*t* = 12.583, 8.934, and 10.033; *P* = 0.011, 0.001, and 0.005) as shown in Table 4.

### 3.4. Comparison of the Disappearance Time of Clinical Symptoms in Two Groups of Patients

As shown in Table 5, compared with the control group, the time to disappearance of clinical symptoms such as fever (2.18 ± 0.01), cough (4.36 ± 1.89), and pulmonary rales (3.86 ± 0.51) in the treatment group was significantly reduced, and the difference was significant (*t* = 7.943, 11.274, and 9.538; *P* = 0.0001, 0.005, and 0.006).

### 3.5. Comparison of Clinical Efficacy between Two Groups of Patients

The cure rate in the treatment group was 76.00% (38/50), which was significantly better than that in the control group (48.00% (24/50)), with a significant difference (*χ*^2^ = 11.724, *P* < 0.001). The total effective rate in the treatment group was 92.00% (46/50), which was significantly better than that in the control group (80.00% (40/50)), with a significant difference (*χ*^2^ = 9.458, *P* = 0.015, Table 6).

## 4. Discussion

Mycoplasma pneumoniae (MP) is one of the common pathogens causing community-acquired pneumonia (CAP) in children. More than 10%-40% of CAP is caused by MP. MP pneumonia (MPP) may develop into life-threatening severe pneumonia in some cases, although it is usually a benign self-limiting disease [5]. As the treatment of choice for MP infections in children, macrolides have been used for MP treatment for many years. However, many clinical isolates of MP cases show resistance to macrolides [6]. However, for the treatment of refractory Mycoplasma pneumoniae in children, the application of immunoglobulin still lacks evidence-based medical evidence.

Mycoplasma pneumoniae is a common pathogen that causes community-acquired pneumonia. In the past, Mycoplasma pneumoniae was sensitive to macrolide antibiotics, and Mycoplasma pneumoniae pneumonia (MPP) was usually a benign self-limiting disease [7]. However, despite appropriate antibiotics, persistent fever and clinical deterioration can lead to severe illness. Two major complications that may be encountered clinically are macrolide-resistant mycoplasma pneumonia and refractory mycoplasma pneumonia [8]. Macrolide-resistant mycoplasma pneumonia manifests with persistent fever and/or no radiographic resolution to macrolide antibiotics and may even develop into severe and complex pneumonia. Tetracycline (doxycycline or minocycline) or fluoroquinolones are alternative treatments for macrolide-resistant mycoplasma pneumonia. Refractory mycoplasma pneumonia is characterized by an excessive immune response to the pathogen [9]. In this context, corticosteroids are considered an immunomodulatory agent for downregulating an overactive host immune response. Macrolide overuse may lead to macrolide resistance, which in turn leads to an increase in macrolide-resistant mycoplasma pneumonia [10].

The host innate and adaptive immune systems work together to combat damage caused by mycoplasma infection. However, the clinical course of pneumonia may worsen when the inflammatory response is overamplified. In refractory mycoplasma pneumonia, the host immune response may lead to lung injury rather than direct microbial damage [11–13]. Therefore, refractory mycoplasma pneumonia is to some extent an immune-mediated disease, and immunosuppressive therapy may therefore be a reasonable approach [14]. Several studies reported the use of immunosuppressive agents, such as corticosteroids or intravenous immunoglobulin, in selected patients. Cell-mediated immunity has been shown to play an important role in the progression of mycoplasma infection [15]. Interleukin (IL) 2, IL8, IL5, IL6, IL18, and other cytokines may be involved in Mycoplasma pneumoniae infection and induce inflammatory response. A high immune response of T cells may lead to the destruction of lung tissue. The immune response produces many inflammatory mediators that may lead to more severe lung damage. Excessive cell-mediated immune and cytokine responses play important roles in refractory mycoplasma pneumonia. Refractory mycoplasma pneumonia is not only an infection but also an immune-mediated disease [16]. Corticosteroids can modulate immunity to inflammatory responses. Corticosteroids have been shown to be effective in improving the clinical manifestations and lung injury of M. pneumoniae infection in children and adults, reducing lung histopathological scores and reducing mortality in severe pneumonia by reducing cytokines and reducing inflammatory responses [17]. Clinical progress has been made in the immunotherapy of refractory mycoplasma pneumonia. Immunoglobulins are considered potent immunomodulators for various immune-mediated diseases, and it has marked activity against Mycoplasma pneumonia and provide additional protection, especially in patients who do not respond well to antibiotic therapy. Immunoglobulins have been reported to be effective in the treatment of many autoimmune and systemic inflammatory diseases [18–20]. Immunoglobulins have significant effects on different immune system effector cells (such as B and T lymphocytes and dendritic cells) and regulate a wide range of genes.

Although only a few studies have reported the use of immunoglobulins in refractory mycoplasma pneumonia, our trial suggests that azithromycin in combination with immunomodulatory therapy is an effective treatment. After treatment in this study, the Th1 (0.16 ± 0.14), Th2 (0.18 ± 0.07), and Th1/Th2 (0.39 ± 0.16) of the study group were compared with those of the control group Th1 (0.37 ± 0.2), Th2 (0.31 ± 0.06), and Th1/Th2 (0.58 ± 0.18), and the decrease was more obvious. Compared with the control group, the immunoglobulin IgG, IgA, and IgM of the study group increased significantly. After treatment, the reduction of inflammatory factors in the study group was more significant than that in the control group. The disappearance time of clinical symptoms and the total effective rate of treatment in the study group were significantly better than those in the control group. The data show that sequential therapy with immunoglobulin combined with azithromycin can effectively improve the cure rate of children with refractory mycoplasma pneumonia. The data analysis shows that the combined medication can significantly shorten the duration of fever in children, improve cough symptoms, promote the absorption of lung inflammation, shorten the hospital stay, reduce the level of inflammatory factors, and regulate the immune system of the body, to achieve the purpose of improving the curative effect.

In conclusion, gamma globulin combined with azithromycin sequential therapy has significant clinical effect in the treatment of children with refractory mycoplasma pneumonia, which can reduce inflammatory factors, improve patients' immunity, and promote disease recovery.

## Figures and Tables

**Table 1:** General information of 2 groups.

Group	Average age (year old)	BMI (kg/m^2^)	Disease duration (d)
Treatment (50)	10.43 ± 1.39	23.81 ± 3.26	6.36 ± 1.56
Control (50)	10.51 ± 1.92	23.31 ± 3.32	6.42 ± 1.59
*t*/*χ*^2^	2.371	3.374	1.856
*P*	0.382	0.593	0.895

**Table 2:** Comparison of Th1, Th2, and Th1/Th2 between the two groups of patients.

Group	*n*	Th1		Th2		Th1/Th2	
		Before	After	Before	After	Before	After
Treatment	50	0.53 ± 0.15	0.16 ± 0.14	0.47 ± 0.13	0.18 ± 0.07	1.41 ± 0.20	0.39 ± 0.16
Control	50	0.57 ± 0.16	0.37 ± 0.21	0.46 ± 0.14	0.31 ± 0.06	1.43 ± 0.15	0.58 ± 0.18
*t*	/	2.019	15.943	1.631	12.055	1.461	13.325
*P*	/	0.245	0.001	0.131	0.005	0.102	0.005

**Table 3:** Comparison of serum immunoglobulin levels before and after treatment between the two groups of patients.

Group	*n*	IgG		IgA		IgM	
		Before	After	Before	After	Before	After
Control	50	8.30 ± 1.60	9.50 ± 1.80	1.20 ± 0.30	1.80 ± 0.40	1.50 ± 0.20	1.60 ± 0.30
Treatment	50	8.50 ± 1.4	11.20 ± 1.60	1.4 ± 0.20	2.20 ± 0.30	1.50 ± 0.30	1.70 ± 0.10
*t*		1.568	12.018	1.064	11.935	1.263	10.881
*P*		0.112	0.001	0.070	0.003	0.065	0.001

**Table 4:** Changes of inflammatory factor levels in patients before and after treatment.

Group	*n*	IL-10		IL-6		IL-2	
		Before	After	Before	After	Before	After
Treatment	50	42.60 ± 6.71	30.20 ± 5.23	85.92 ± 5.20	40.52 ± 2.83	67.80 ± 6.31	30.61 ± 1.50
Control	50	41.52 ± 5.90	19.91 ± 5.40	85.71 ± 4.93	48.21 ± 3.80	65.62 ± 2.84	21.20 ± 2.41
*t*		1.532	12.583	1.202	8.934	2.075	10.033
*P*		0.596	0.011	0.840	0.001	0.940	0.005

**Table 5:** Comparison of the disappearance time of clinical symptoms in the two groups of patients.

Group	Fever	Cough	Pulmonary rales
Control (*n* = 50)	4.28 ± 1.33	6.27 ± 1.57	5.86 ± 0.57
Treatment (*n* = 50)	2.18 ± 0.01	4.36 ± 1.89	3.86 ± 0.51
*t*	7.943	11.274	9.538
*P*	0.001	0.005	0.006

**Table 6:** Comparison of clinical efficacy between the two groups of patients.

Group	Healing	Show effect	Effective	Ineffective	Total effective	Total efficiency
Treatment (*n* = 50)	16 (32.00)	22 (44.00)	8 (16.00)	4 (8.00)	38 (76.00)	46 (92.00)
Control (*n* = 50)	10 (20.00)	14 (28.00)	16 (32.00)	10 (20.00)	24 (48.00)	40 (80.00)
*χ* ^2^	/				11.724	9.458
*P*	/				<0.001	0.015

## Data Availability

All data was provided in the manuscript.
